The article "Application of Image Processing Technology in the Diagnosis of Football Injury" was retracted in 2023. Reasons: signs of a paper mill; suspected computer-generated content; unreliable results or conclusions; concerns about the data.

# Application of Image Processing Technology in the Diagnosis of Football Injury

**DOI:** 10.1155/2022/5926098

**Published:** 2022-08-05

**Authors:** Liyun Xu, Zhubo Xu

**Affiliations:** Physical Education Department, Anhui University of Finance and Economics, Bengbu, 233041 Anhui, China

## Abstract

With the hot development of football, sports injuries caused by football have also received special attention. In football games, although there are medical staff on and off the field always on call to protect the safety of players, because of the complexity of diagnosis work, medical staff can easily lead to diagnostic errors due to factors such as fatigue, which seriously affects the condition of athletes. Image processing is a technology that uses computer to process images, which can greatly overcome the uncertain factors brought by manual diagnosis. Based on this, this paper uses image processing technology and pattern recognition as technical means to explore the specific application of image processing in football injury diagnosis. This paper firstly takes football clubs as the main research object and analyzes and explores the specific utility of image segmentation and feature recognition in sports injury image processing. Then, starting from the relevant image features, the paper analyzes and compares the sensitivity of support vector machine pattern recognition and neural network pattern recognition in football injury diagnosis. This article comprehensively summarizes the application of image processing technology in the diagnosis of football injuries and puts forward constructive suggestions for its subsequent development. Experiments show that the effect of pattern recognition is often different for different injury parts of football. Among them, the sensitivity of pattern recognition based on image processing can reach 68.9%, and the detection rate of football injuries can also be maintained at about 81.2%. This fully shows that image processing technology can play an active role in the actual football injury diagnosis, and provide very valuable information for clinical diagnosis.

## 1. Introduction

With the advancement of medical level, the diagnosis of football player injuries has become more and more refined, but this method of diagnosis often brings high time-consuming and high cost. Moreover, in the diagnosis process of this mode, the diagnosis work often needs to go through a lot of steps and processes, which brings a great burden to the medical staff. At the same time, the traditional clinical diagnosis still relies on the physician's own experience and related abilities, which brings a lot of uncertain factors to the diagnosis of football injuries, and leaves a great physical hidden danger. Image processing is a brand-new processing mode derived from computer. Its combination with football injury diagnosis can buy a lot of time for athletes' injury diagnosis and make adequate preparations for subsequent clinical diagnosis. On this basis, image processing can provide a lot of injury feature information for sports injury diagnosis and provide rich data support for subsequent diagnosis. At the same time, this move can also summarize the experts' experience in diagnosing sports injuries and provide a reference for the establishment of an auxiliary diagnostic system. In addition, image information can often break the limitations of time and space, which also provides a corresponding platform for telemedicine diagnosis and treatment. Image processing technology can also build a perfect diagnosis and treatment model.

Sports injury is an unavoidable problem during exercise, and timely injury diagnosis is the best way to protect the health of athletes. Waterworth et al. conducted a study of senior football clubs in the Scottish Borders to analyse the effects of physiotherapy and chemical therapy in football injuries. Among them, physiotherapists and chemical therapists visit the club once a week, and they are allowed to obtain information on all new or recurring injuries that arise during games or football-related training [1]. Kullak-Ublick et al. aim to determine the incidence and patterns of injuries in football players and the associated consequences and labor losses in everyday life. They recorded injury rates by age group during games, collected data on the occurrence and consequences of injuries, and found that serious football injuries account for the largest share of all injuries [2]. Araki et al. pointed out that spikes can cause serious lacerations in football, but the incidence of these injuries is unclear. Therefore, in order to study its incidence, they collected data on serious tear injuries in amateur and professional football players and established a digital scale based on this [3]. Haddad et al. pointed out that in medical care, a specific way of diagnosing an injury is neither specific nor predictive of the patient's subsequent clinical course. So they designed a simple diagnostic aid system based on computer. During the experiment, the system relies on related algorithms to connect various medical machines in series to finally achieve the timeliness of diagnosis [4]. The above experts and scholars have analyzed the methods of sports injury diagnosis from different angles, but the methods they propose are either difficult to implement, or have high operating costs and long time, which cannot meet the timeliness and urgency of football sports injury diagnosis.

Image processing technology is simple to operate and does not require high consumption. In recent years, more and more scholars have carried out research on image processing technology. Kamel et al. pointed out that image processing-based computed tomography planes can provide a powerful assessment of liver problems, early detection of neovascularization, and tumor staining. Compared with conventional methods, computer imaging platforms based on image processing techniques can better assess tumor burden. In addition, they pointed out that the platform can accurately delineate the anatomy of liver vessels for segmental localization and assist in surgical and nonsurgical planning [5]. Apraites et al. faced great challenges in processing 10,000 images. In order to convert these image data into useful data information, they developed an automatic image processing system based on image processing technology. At the same time, they also described some key techniques for reading the imaging protocol and processing images [6]. Wu et al. proposed a method to speed up various image processing operations. During his research, he used a fully convolutional network trained on input-output pairs that exhibited operator actions. After training, the original operator does not need to run at all, and the trained network runs at full resolution and in constant time. Finally, they study the impact of network structure on approximation accuracy, running time, and memory footprint and identify specific structures that balance these considerations [7]. Cheung et al. pointed out that light field imaging has become an emerging image processing technique that can capture richer visual information from our world. Different from the traditional processing technology, the general image processing only does the two-dimensional projection of the light in the scene in the angular domain; the light field collects light from all directions and multiplexes the angular domain information lost in the transmission method [8]. The above experts and scholars analyzed the application of image processing technology from different angles, but they did not study the practical application of image processing in sports injuries.

After a series of experiments and analysis, we can know that in the process of football, athletes' limbs are often the most vulnerable to injury, accounting for 78.25% of athletes' injuries. Among them, among limb injuries, athletes' legs and leg joints are often the most vulnerable parts, accounting for 23% and 36% of injuries, respectively. With the help of image processing technology, the detection rate of common injuries such as strain can be basically maintained at 63%, which can meet the actual needs of clinical diagnosis. In addition, for joint injuries and bone injuries, for example, the injury detection rate can also be maintained at about 81.2%, which can more accurately identify and detect different types of injuries. This fully shows that medical staff based on image processing technology can diagnose the disease at the first time and can ensure the accuracy of diagnosis to a large extent. On this basis, the combination of image processing technology and sports injury diagnosis has great practical significance and application value.

## 2. Image Processing Technology and Football Injury Diagnosis

### 2.1. Diagnosis of Football Injuries

Football is one of the most popular sports at present, and it has attracted a large number of loyal people. However, in the process of intense sports, injuries are inevitable due to collisions between players on both sides [9]. Also, due to different impacts and angles, football players are injured at different locations and to the same extent. When faced with an injured athlete, prompt and accurate treatment and diagnosis are imperative [10]. Sports injuries are not only a concern for athletes but also a concern for healthcare workers. On the one hand, different degrees of sports injuries will bring different degrees of potential hidden dangers to athletes, seriously endangering football players' careers on the field. On the other hand, diagnosing and treating sports injuries is a very long period of practice, which will directly affect a series of athletes' training and competition. In this environment, how to solve the problem of sports injuries is another difficult problem before us. Moreover, clinical sports injury diagnosis often fails to obtain corresponding results in a timely manner, which also causes a great psychological burden to football players [11]. The current flow of injury diagnosis and treatment used in football is shown in Figure 1.

In the process of injury diagnosis in this model, the medical and nursing staff first collects the characteristics of the injury surface of the athlete to find the external manifestations and characteristics corresponding to the injury. After obtaining the relevant characteristics, if the injury surface of the athlete is not particularly serious, then the athlete can be directly diagnosed and judged at this time, and then, the result of the diagnosis and clinical treatment can be obtained according to the judgment. However, if there are many parts involved in the damage surface, it is necessary to assist other inspections to judge the actual situation of the damage. After comprehensively judging these injuries, medical staff can identify the results of the injury judgment according to clinical experience and then finally get the diagnosis results and carry out treatment [12]. However, in this process, we also found that the judgment and diagnosis of injury are often based on the experience of medical staff, and related auxiliary inspection equipment often cannot directly obtain results, which may delay the optimal treatment time for injury.

In the process of football injury diagnosis, we generally use the etiological diagnosis methods such as inspection, palpation, and auscultation. In this diagnosis mode, the diagnosis is often based on the self-cultivation of medical staff. But in this process, because football players have already faced huge injuries, this process may be accompanied by intense pain [13]. Therefore, at this time, the relevant inquiries or the etiological diagnosis of the athletes will bring great errors.

### 2.2. Image Processing Technology

Image is the most capable of conveying information and data carrier, which is an important basis of human vision and machine vision [14]. In the process of diagnosing injuries in football players, images are an important tool for recording live and real-time data. In this process, the role of the image is that it can observe the football player's injury signal through a variety of measurement and detection peripherals and then obtain the most realistic data [15]. At the same time, the transmission of damage information through images can ensure the integrity of the required information, and it is not easy to be disturbed by the external environment. Therefore, it is of great significance to use images for damage description.

Image processing is a kind of computer technology, which mainly includes image segmentation and image recognition. In the process of image processing of football injuries, image processing can separate the injured part from the healthy part, so that relevant experts can only focus on observing the injured part of the athlete. Secondly, image processing can also identify the characteristics of the injury on the basis of the athlete's injury, to help the medical staff to accurately judge the type of injury and prescribe the right medicine based on this [16]. Image processing technology has many applications in the diagnosis of sports injuries. In addition, there are many other links in image processing, which are also widely used in many fields. The basic application fields of image processing technology are shown in Figure 2.

Image processing technology is now widely distributed in various fields, including aviation technology and biomedicine. In the process of image representation of football injuries, we fully exploited the utility of image processing technology in the diagnosis of actual football injuries [17]. In this process, the computer collects and stores relevant information through external devices such as cameras. A series of means of image acquisition and editing, information acquisition and transmission, data storage, and other operations are realized by digital means. Among them, the operation of image editing specifically includes flattening, cropping, resolution adjustment, and damaged image repair or restoration. Image cutting is carried out on the basis of image editing. First, the target elements need to be retrieved, and then, they are sorted and classified according to their characteristics, so that an image model and a database for storing image information can be constructed. On the basis of the database, the relevant staff can integrate all the data to improve the processing efficiency. In this actual operation process, the image acquisition and acquisition of football injury will also be carried out according to the above steps. In order to make the above process conform to the running habits of the computer, we abstract and integrate it into a series of processing processes. The basic process of image processing of football injuries is shown in Figure 3.

From the above, we can basically know that in the basic process of football injury image processing, the first thing we need to do is to acquire the athlete's injury image and then preprocess the image on this basis [18]. Next, this paper will focus on analyzing the basic process of football injury image processing.

- Image acquisition

Image acquisition is the process of collecting images of football players in live games or training, which is the first step in our analysis of football injuries and diagnosis. In the acquisition process, because football players are often in high-speed motion, the generally selected acquisition tools are high-speed cameras or video cameras. Although the image can only reflect the scene at a certain moment, it also reproduces the three-dimensional scene, so this is also the basis for us to use the captured image to replace the real scene. After obtaining the relevant image information, we can directly transfer the data to the computer, thus saving a lot of time. In the process of acquiring sports injury images, timely and efficient data transmission is the premise and guarantee of timely diagnosis.

(ii) Preprocessing

In the image acquisition stage, we have collected a large number of images or videos. However, due to the differences in the field environment and equipment, the collected images cannot be directly used by the computer [19]. Therefore, before this, we need to preprocess the image to eliminate unnecessary interference information of the image. In the process of image processing, due to various processing methods, we need to process images according to actual needs. In the process of football injury image processing, what we need to pay attention to is the difference of color and the distortion of graphics.

(iii) Image segmentation

After preprocessing the football injury images, we can basically get ideal images that meet the requirements. However, in an ideal image, there are many areas with different characteristics, which is not conducive to the transmission of image information and the later image processing. The segmentation of football injury images can separate the characteristic regions and then extract the main research objectives from them, reducing unnecessary workload. However, the actual segmentation of football injury images is not very easy, and the segmentation effects are often not the same. For example, the segmentation of the image of the automobile assembly line can be divided into the background area and the workpiece area and can also be divided into the staff area and the nonstaff area. In recent years, neural network methods have made good progress in the field of image segmentation, which will promote the continuous development of image segmentation implementation.

(iv) Feature recognition and classification

After completing the segmentation of sports injury images, we can obtain several regions with different characteristics. However, in these regions, due to the obvious differences in features, it is impossible to completely distinguish them by relying solely on the human eye [20]. Feature recognition is a general term for distinguishing and classifying features of images. Generally speaking, feature recognition and classification have a lot in common, so often after feature recognition is completed, the category of features is very clear. For example, in industries such as manufacturing or security, after identifying the characteristics of an image, its type and category are naturally differentiated. In the process of sports injury recognition, we are gradually forming image recognition methods with neural networks as the mainstream, such as convolutional neural networks, regression neural networks, and other methods with superior performance.

(v) Positioning and diagnosis

After the classification and feature identification are clear, the most critical is positioning and diagnosis. In the process of football injury diagnosis, the first thing we need to do is to find the injury point, and the process of finding the injury point is the process of positioning. Locating damage points is based on feature identification and classification. On the one hand, we can reduce unnecessary searching and searching through feature matching. On the other hand, through feature classification, we can preferentially search for the same feature segment, thereby saving time and saving plenty of time for later diagnosis.

So far, we have briefly sorted out the basic process of football injury image processing. In this process, we realize the combination of image processing technology and football injury diagnosis from a theoretical point of view. However, medical diagnosis often involves many verifications or tests, so the article will analyze the entire process of combining the two from a mathematical point of view.

From a mathematical point of view, after preprocessing the image of sports injury, we can get a more ideal digital image of sports injury, but the areas of various meanings are intertwined in the image, and it is impossible to provide people with a simple and clear damage area. Sports injury image segmentation can help medical staff to qualitatively analyze the injured tissue and improve the accuracy of medical staff in diagnosing football sports injuries. The image segmentation of football injuries is as follows:

(1) $$\begin{array}{c} G_{r}=M-f\left(x,y\right)-B\left(d,\rho \right), \end{array}$$

(2) $$\begin{array}{c} f_{\text{or}}{\left(x,y\right)}^{T}=f_{pr}\left(x,y\right). \end{array}$$

In the above formula, *G*_*r*_ represents the preprocessed image of football injury, and *M* and *B*, respectively, represent the color channel value in the athlete's injury image. Through this formula, we can basically realize the color distinction and basic recognition of the preprocessed image. Next, we perform type of *f* transformation operations on pixel (*x*, *y*) in the image and then implement image segmentation.

After the image is segmented, the graphic features of the image become more and more obvious, so we can perform damage feature extraction on it. The mathematical expression of feature extraction is:

(3) $$\begin{array}{c} \omega =\max\left(\sum f_{pr}\left(a,b\right)\right), \end{array}$$

(4) $$\begin{array}{c} H=\max\left(\overset{M}{\underset{i=1}{\sum }}f_{ab}\left(\omega ,B\right)\right)-\min\left(\overset{M}{\underset{i=1}{\sum }}f_{\omega }\left(a,B\right)\right), \end{array}$$

(5) $$\begin{array}{c} T=\frac{A}{\omega \times H}\tan\frac{\left(a-b\right)}{B}. \end{array}$$

Among them, *ω* represents the maximum width of the football injury in the image, *H* represents the maximum height of the football injury in the image, and the two together constitute the overall graph *T* of the football injury image.

After image segmentation and feature extraction, the characteristics of football injury images are becoming more and more obvious, which has met the requirements of related data training. On this basis, we train on a series of processed sports injury images to fit the subsequent pattern recognition process. Next, we perform image recognition on sports injuries, and the formula is as follows.

(6) $$\begin{array}{c} F=1-\frac{4\pi A}{T^{2}}, \end{array}$$

(7) $$\begin{array}{c} D=\overset{n}{\underset{j=1}{\sum }}\frac{1}{1+4\pi A{\left(i+1\right)}^{2}}\rho \left(i,j\right). \end{array}$$

In the above formula, *F* represents the sensitivity of football injury recognition, which is mainly affected by the overall graph. Among them, *D* represents the accuracy in the process of pattern recognition, which depicts the gap between the image and the actual sports injury.

Based on the above, we have basically realized the acquisition, segmentation, and feature recognition of football injury images. On the basis of the above images, we use support vector machine and BP neural network to train the above image data and then initially realize the recognition of support vector model based on image processing. In the specific operation process of football injury diagnosis, the image processing unit is connected with the digital image information of the football match scene. Once a sports injury problem occurs, medical staff can immediately retrieve relevant image information to diagnose injuries in football. However, whether pattern recognition based on image processing technology can play its due role in the process of football injury diagnosis still needs to be further tested by our experiments.

## 3. Recognition of Sports Injury Patterns Based on Image Processing

The images collected in this study are from professional football clubs, in which the sports injuries of football players are the first-hand images obtained directly in scene monitoring using digital cameras and high-definition digital cameras. At the same time, in order to ensure the quality of the pictures, the images are stored in the computer in JPG format. In order to reduce the interference caused by the outside world, we use image processing software to remove some irrelevant backgrounds and normalize the image; its size is 256 × 256. Through the acquisition and analysis of the above data, we can find that football injuries often show different characteristics in different parts, and the injuries in different parts will also affect the final diagnosis. In order to further analyze the specific situation of football injuries, we analyzed the diagnosis of different parts of football injuries and the distribution of football injuries. The results are shown in Table 1 and Table 2, respectively.

The above data shows that in the process of football, athletes' limbs are often the most vulnerable to injury, accounting for 78.25% of athletes' injuries. Among them, among limb injuries, athletes' legs and leg joints are often the most vulnerable parts, accounting for 23% and 36% of injuries, respectively. However, injuries to the head and internal organs of athletes tend to be more serious than the limbs, and the diagnosis is often extremely dangerous.

Therefore, in intense football sports, it is particularly important to ensure the physical safety of players and to identify and diagnose their injuries in a timely manner. With the support of the above data, we use support vector machine to identify and train different damage pictures and ensure the integrity of the pictures as much as possible. At the same time, in order to further improve the accuracy of pattern recognition, we also added BP neural network for recognition and comparison. Among them, the pattern recognition under different damaged parts is shown in Table 3.

Table 3 shows that different parts have different recognition situations after a series of training and recognition. Among them, the pattern recognition rate of SVM for head damage is 45.11%, while the recognition rate of BP neural network is basically 36.17%. In further contrast, we found that the damage recognition rates for the waist and legs were relatively high, reaching 69.23% and 66.36%, respectively. This shows that for different injury sites, different pattern recognition has its own characteristics. In the above analysis process, we selected several pictures for different damaged parts, and then used the pattern recognition algorithm to judge and simulate the diagnosis. The damage judgment in different modes is shown in Table 4.

Table 4 shows that for the same 200 images, the error rates of different pattern recognition methods are often different. Among them, the number of wrong pictures for SVM pattern recognition is 13, and the number of BP pattern recognition is 11. In contrast, based on image processing technology, the judgment of damage is greatly improved, the error rate of SVM is basically 6.5%, and the error rate of BP neural network is 5.5%.

## 4. Recognition Results of Football Injury Patterns

On the basis of the data collected above, we have a general understanding of damage recognition in different parts and modes. Image processing provides technical support for us to better diagnose and discover the hidden dangers behind football player injuries. In this case, by matching different pattern recognition algorithms, we will be able to get more accurate player injuries. Among them, the recognition sensitivity of different modes for different injury parts of football is shown in Figure 4.

Figure 4 shows that the effect of pattern recognition tends to be different for different injury sites. Among them, there is a big difference between the two patterns of torso injury recognition. The pattern recognition sensitivity based on SVM can reach 68.9%, but the recognition sensitivity based on BP is only 64.3%. Moreover, for intrinsic damage such as nerves, pattern recognition only relying on image processing technology often cannot achieve ideal results, and the average recognition sensitivity of the two is only 56%. This shows that only sensitive identification and efficient diagnosis of some damaged parts can be achieved by relying on image processing technology.

The sensitivity of diagnosis is an important indicator to measure pattern recognition. In addition, the error rate of diagnosis is also one of the indicators that can reflect the effect of pattern recognition. In the process of football injury identification, if there is an error, it will directly affect the timely treatment of the athlete and even life-threatening in serious cases. Therefore, it is necessary for us to comprehensively evaluate the error rate. Among them, the error rate of football injury recognition is shown in Figure 5.

Figure 5 shows that, after many experiments, the recognition error rate of football injuries continues to decrease, gradually showing the characteristics of low speed. Among them, in the first three experiments, the pattern recognition based on SVM has always maintained a relatively low error rate, and the comprehensive error rate does not exceed 8.5%. In particular, in the last three experiments, the pattern recognition error rate showed a linear downward trend, with the lowest error rate reaching 7.1%.

The error rate only describes the errors in the identification process, but in the actual identification process, it is necessary to accurately detect the specific injury type, so as to provide first-hand information for clinical diagnosis and provide conditions for further treatment. Therefore, it is necessary to study the specific conditions of injuries in different parts of football, in which the detection rates of different parts are shown in Figure 6.

Figure 6 shows that the detection rate of injuries in different parts of football is often restricted by many factors. Among them, the detection rate of common injuries such as strain can be basically maintained at 63%, which can meet the actual needs of clinical diagnosis. In addition, for joint injuries and bone injuries, for example, the injury detection rate can also be maintained at about 81.2%, which can more accurately identify and detect different types of injuries. However, we also found that if the athlete had more than one injury at a time, the detection rate in this mode would be directly affected.

## 5. Conclusion

The combination of image processing technology and pattern recognition provides a practical reference for football injury diagnosis. Starting from the general sports injury diagnosis methods, this paper first analyzes the individuality and commonality of these methods, then reveals the shortcomings of these methods, and gradually transitions to the image processing technology. Then, this paper focuses on analyzing the specific functions of image segmentation, image feature recognition, and other technologies in the diagnosis of football injuries. Finally, combined with the method of pattern recognition, this paper takes SVM and neural network as examples to analyze the application of image processing technology in the actual process of football injury diagnosis. Experiments show that image processing technology can greatly improve the sensitivity and accuracy of football injury diagnosis. However, due to time reasons, this paper does not consider the selection of eigenvectors. In the future, this paper will further analyze the influence of feature vector difference on the final result of image processing to make up for the lack of the paper.

## Figures and Tables

**Figure 1:** The diagnosis process of football injuries.

**Figure 2:** Application areas of image processing technology.

**Figure 3:** Image processing flow of football injuries.

**Figure 4:** Recognition sensitivity of different injury sites in football.

**Figure 5:** Error rate of football injury identification.

**Figure 6:** Detection rate of injuries in different parts of football.

**Table 1:** Diagnosis of different injury sites in football.

Injury site	Damage ratio	Recognition rate	Diagnosis
Limbs	78.25	88.12	Mild
Trunk	9.9	76.21	Moderate
Head	7.25	61.20	Severe
Internal organs	3.41	45.91	Severe

**Table 2:** Distribution of football injuries.

Injury site	Damage ratio	Damage distribution
Head	11	6.7
Shoulder	7	4.2
Wrist	8	4.5
Waist	9	4.9
Legs	23	11.3
Leg joints	36	21.8

**Table 3:** Pattern recognition at different injury sites.

Injury site	SVM	BP	Other
Head	45.11	36.17	36.21
Shoulder	57.6	54.22	45.91
Wrist	58.2	54.15	56.11
Waist	69.23	64.19	59.91
Legs	66.36	61.31	56.21
Leg joints	59.98	51.28	48.45

**Table 4:** Damage judgment in different modes.

Mode	Total	Correct number	Number of errors	Failure rate
SVM	200	187	13	6.5
BP	200	189	11	5.5
Original	200	156	44	22
Other	200	161	39	19.5

## Data Availability

No data were used to support this study.
